This article has been retracted.

# Evaluation of a Novel Quality of Life Scale for Schoolchildren with Nonstrabismic Binocular Vision Anomalies

**DOI:** 10.1155/2020/4723402

**Published:** 2020-07-30

**Authors:** Jiali Hu, Guokun Wang, Zhe Zhou, Yan Sun, Qingling Zhang, Jinhui Wu, Yu Gao

**Affiliations:** ^1^Department of Ophthalmology, Hongkou Branch of Changhai Hospital, Naval Medical University, Shanghai 200081, China; ^2^Department of Ophthalmology, Eastern Hepatobiliary Surgery Hospital, Naval Medical University, Shanghai 200433, China; ^3^Department of Cardiovascular Surgery, Changhai Hospital, Naval Medical University, Shanghai 200433, China; ^4^College of Science, Hohai University, Nanjing, 210098 Jiangsu, China

## Abstract

**Background:**

The professional Quality of Life Scale (QLS) can provide a valuable reference for the diagnosis of visual function anomalies. In the present study, we aimed to design a novel QLS to specially quantify the life quality of schoolchildren with nonstrabismic binocular vision anomalies (NSBVAs) in China.

**Methods:**

The novel QLS, named QOL-CVF20, was established based on classical vision-related scales and the administration of the questionnaire to 116 schoolchildren with NSBVAs and 100 healthy schoolchildren in China. The diagnostic reference value between QOL-CVF20 and VF-14 was evaluated on the questionnaires to 240 schoolchildren with NSBVAs and 238 healthy schoolchildren.

**Results:**

All the subjects could complete the QOL-CVF20 questionnaires independently. QOL-CVF20 had good structural validity, content validity, and discriminant validity, when it was applied in Chinese schoolchildren. The average score of the NSBVA group was significantly lower than that of the control group (49.0 ± 6.9 vs. 69.7 ± 6.7, respectively; *P* < 0.01). Moreover, the average score of cured NSBVA schoolchildren after treatment (61.8 ± 22.6) was significantly improved (*P* < 0.01). Receiver operating characteristic curve analysis showed that QOL-CVF20 reflected strong separation between the NSBVA and healthy groups (AUC = 0.901). Meanwhile, QOL-CVF20 could detect individuals with NSBVAs with specificity of 0.847 and sensitivity of 0.846. The critical value of 58.50 in QOL-CVF20 could be effectively applied for quality of life assessment in schoolchildren with NSBVAs.

**Conclusions:**

QOL-CVF20 could quantify the life quality of schoolchildren with NSBVAs and might be served as a valuable reference for early diagnosis and clinical evaluation of NSBVAs.

## 1. Introduction

Today, binocular vision anomalies are important factors affecting children's cognitive development and educational progress [1]. Nonstrabismic binocular vision anomalies (NSBVAs), a potential loss of binocular vision, might be the intermediate state between normal binocular vision and strabismic binocular vision anomalies [2, 3]. With the popularity of the computer, mobile phone, and other video terminals, it has been reported that NSBVAs are highly prevalent among schoolchildren [4, 5]. Currently, the diagnosis of NSBVAs is mainly based on the description of clinical signs. However, there are certain differences between doctors' assessment and children's subjective description. Therefore, the early diagnosis and treatment of NSBVAs could not be implemented well.

With the development of medical research and health concepts, the medical model has evolved from simple biomedicine to a biopsychosocial pattern [6]. The quality of life has gradually been introduced into the field of medical research and has become an index system for evaluating health and clinical efficacy. Quality of life mainly focuses on the subjective experience of the patients but is not an objective evaluation of the functional state of the bodies [7]. Patients with NSBVAs often suffer from varying degrees of quality of life, such as adjustment and convergence anomalies and eye symptoms including discomfort, pain, headache, blurred vision, visual fatigue, double images, word skip, or line skip [8]. Due to the uniqueness of schoolchildren's physiology and psychology, it is urgent to establish a quality of life evaluation system specifically for schoolchildren.

The Quality of Life Scale (QLS) has been increasingly used as an important measure in medical and philosophical literatures. The professional QLS can provide a valuable reference for early diagnosis and clinical evaluation of many diseases [9, 10]. Currently, several vision-related QLS had been applied in the clinic, including the WHO Quality of Life questionnaire (WHOQOL-100), 14-item Vision Function questionnaire (VF-14), and 25-item National Eye Institute Visual Function Questionnaire (NEI VFQ-25) [11–13]. VF-14 was developed by Steinberg in 1994, originally for visual function assessment in cataract patients. After the improvement by Linder in 1999, VF-14 has been widely used to assess visual impairment in patients with various eye diseases [14, 15]. However, there is no professional QLS severed for NSBVA diagnosis in schoolchildren until now.

In the present study, a novel QLS, named QOL-CVF20, was designed to specially quantify the life quality of Chinese schoolchildren with visual function anomalies. Based on a retrospective study, the application of QOL-CVF20 on health and clinical efficacy in schoolchildren with NSBVAs was evaluated. QOL-CVF20 could provide important references and assistance for the early diagnosis of NSBVAs in schoolchildren.

## 2. Materials and Methods

### 2.1. Study Population

Schoolchildren with NSBVAs were diagnosed in the Department of Ophthalmology of Changhai Hospital from July 2013 to August 2017. Diagnosis of NSBVAs was made by the comprehensive analysis of abnormal binocular vision symptoms (eye discomfort and swell, blurred vision, visual fatigue, complex image, text skipping or overlap, etc.) according to Morgan normal values and Sheard's or Percival's criterion. The patients with strabismus, amblyopia, organic eye disease, and other general anomalies were excluded. Schoolchildren aged 8-10 who were capable of understanding the content of the Chinese-language questionnaires correctly were enrolled in this study. This study was carried out in accordance to the principles of the Declaration of Helsinki and approved by the Medical Ethics Committee in Changhai Hospital. All the children's parents or legal representatives accepted the study's participation principles and signed an informed consent.

### 2.2. Establishment of QOL-CVF20

Based on the classical vision-related QLS (WHOQOL-100, VF-14, and NEI-VFQ25) [11–13], a quality of life Chinese questionnaire containing 20 items (QOL-CVF20) was established for visual function anomaly diagnosis in schoolchildren. In order to facilitate the schoolchildren's understanding, 5 easy-to-distinguish frequency adverbs (always, often, sometimes, rarely, and never) were selected as the answer options (Supplemental data Table S1). There were 4 domains in QOL-CVF20, which were binocular visual function domain (items 1-10), self-care ability domain (items 11-13), activity communication ability domain (items 14-16), and psychological domain (items 17-20).

### 2.3. Implementation of QOL-CVF20

All the subjects should independently complete the QOL-CVF20 questionnaires under the guidance of investigators. The answer options (always, often, sometimes, less, and never) were recorded as specific scores. From item 1 to item 12, always = 1, often = 2, sometimes = 3, less = 4, and never = 5. From item 13 to item 20, always = 5, often = 4, sometimes = 3, less = 2, and never = 1. The summation of all items' scores was calculated as the total score of QOL-CVF20.

### 2.4. Determination of Minimum Sample Size

The minimum sample size was identified according to the sample capacity formula of reliability test (*n* = [(*Z*(*α*)/2)/(*Z*(*R*) − *Z*(*R* + CI_*H*_))]^2^ + 3). In this formula, *n* represented the sample size, *R* represented the reliability, and CI_*H*_ represented the half width of the confidence interval of overall reliability. *Z* represented the Fisher *Z* transformation, that is, *Z*(*R*) = (1/2)ln((1 + *R*)/(1 − *R*)). Taking *α* = 0.05, *R* = 0.70, and CI_*H*_ = 0.05, the minimum sample size was calculated as *n* = 89.

### 2.5. Statistical Analysis

All statistical analyses were performed by SPSS version 22.0. Quantitative variables were presented as mean ± SD. Two-tailed Student *t*-test and paired-sample *t*-test were used for statistical comparison of the continuous variables. Univariate linear regression analysis was applied to identify the correlation between QOL-CVF20 and VF-14. Receiver operating characteristic (ROC) curves were established for validity prediction analysis between QOL-CVF20 and VF-14. *P* values less than 0.05 were considered statistically significant.

## 3. Results

### 3.1. Parametric Analysis of QOL-CVF20

A total of 116 schoolchildren with NSBVAs and 100 healthy schoolchildren were enrolled from July 2013 to February 2015. All subjects could complete the QOL-CVF20 questionnaires within 19 min, with an average time of 15.5 ± 2.4 min. The recovery rate of scale was 100%, and the overall efficiency was 92.6%. Invalid questionnaires were due to unanswered entries, which were mainly located in items 17 and 20.

The related parametric of QOL-CVF20 was analyzed based on 109 valid questionnaires from the NSBVA group and 91 valid questionnaires from the control group. As shown in Table 1, the maximal coefficient of variation was 49.74% (item 11), while the minimal coefficient of variation was 39.69% (item 8). Calculated with the total score, the highest correlation coefficient was 0.60 (item 2) and the minimum was 0.30 (item 11). The correlation coefficients between each item score and total score had significant differences (all *P* < 0.01). The Kaiser-Meyer-Olkin (KMO) test demonstrated that the original variable was suitable for factor analysis (KMO = 0.81). Then, 4 common factors (F1, F2, F3, and F4) were extracted based on the principles of eigenvalues greater than 1. The cumulative variance contribution rate was 53.15% (Figure 1). Items 1-10 (F1 > 0.5) belonged to the binocular visual function domain, items 17-20 (F2 > 0.5) belonged to the psychological domain, items 11-13 (F3 > 0.5) belonged to the self-care ability domain, and items 14-16 (F4) belonged to the activity communication ability domain (Table 1). All the items were confirmed to be closely related to the total score by stepwise regression analysis, and items 1-10, 13, 19, and 20 were identified to contribute to distinguish NSBVAs by stepwise discriminant analysis (Table 1).

### 3.2. Validity Evaluation of QOL-CVF20

Content validity analysis showed that all the correlation coefficients between the item score and the corresponding domain score in QOL-CVF20 were greater than 0.55 (Table 1). The maximum correlation coefficient was 0.85 (item 11), while the minimum correlation coefficient was 0.56 (item 4). The correlation coefficients between the 4 domain scores and total score had significant differences (*r* = 0.84, 0.48, 0.49, and 0.54, respectively. All *P* < 0.01). The results showed that QOL-CVF20 had a good content validity.

According to the QOL-CVF20 result, the average score of the NSBVA group (49.0 ± 6.9, *n* = 109) was significantly lower than that of the control group (69.7 ± 6.7, *n* = 91, *t* = −21.41, *P* < 0.01; Table 2). After 2-6-month treatment training, 88.8% of the NSBVA patients (113/116) were cured and had no regression during the 3-month follow-up. A total of 86.7% of questionnaires (98/113) were identified as valid for the QOL-CVF20 survey. The average score of the cured group (61.8 ± 22.6, *n* = 98) was significantly higher than that of the NSBVA group (49.0 ± 6.9, *n* = 109, *t* = −5.63, *P* < 0.01; Table 3). The results showed that QOL-CVF20 had a good discriminant validity.

### 3.3. Reliability Evaluation of QOL-CVF20

The 116 patients with NSBVAs received a 2^nd^ survey of QOL-CVF20 at 2 weeks after the 1^st^ survey. The average score of 112 valid questionnaires was 48.9 ± 6.7. No significant difference (*t* = 1.97, *P* > 0.05) and no significant correlation (*r* = 0.98, *P* < 0.01) were found between the 1^st^ and 2^nd^ surveys. The results showed that QOL-CVF20 had a high crosstime consistency. Internal consistency reliability showed that all the 4 domains of QOL-CVF20 had good reliability (*α* = 0.85, 0.75, 0.71, and 0.73, respectively). Based on valid questionnaires from the 1^st^ survey, the average score of odd items was 34.9 ± 4.0, and the average score of even items was 34.8 ± 3.9. No significant correlation was found between the two sets of items (Rh = 0.78, *P* < 0.01). Split-half reliability showed that QOL-CVF20 had a high crossindicator consistency (*R* = 0.88).

### 3.4. Responsiveness Evaluation of QOL-CVF20

A total of 93 questionnaires from cured NSBVA schoolchildren were identified valid in both before and after treatment. The average score of the cured group (61.4 ± 23.0) was significantly higher than that of the untreated group (49.7 ± 7.2, *t* = 5.09, *P* < 0.01). The effect size (ES) analysis proved that QOL-CVF20 had a moderate effect on the changes in clinical symptoms (ES = 0.53, Table 4).

### 3.5. Comparative Analysis between QOL-CVF20 and VF-14

Both QOL-CVF20 and VF-14 were provided to 240 schoolchildren with NSBVAs and 238 healthy schoolchildren from March 2015 to August 2017. The total effective response rate of QOL-CVF20 was 91.21% (221 valid questionnaires from the NSBVA group and 215 valid questionnaires from the control group), while the total effective response rate of VF-14 was 89.54% (217 valid questionnaires from the NSBVA group and 211 valid questionnaires from the control group). No significant difference was found on the effective response rate between the scales of QOL-CVF20 and VF-14 (*P* > 0.05).

A total of 423 questionnaires were identified valid both in QOL-CVF20 and in VF-14 (215 schoolchildren with NSBVAs and 208 healthy schoolchildren). According to the QOL-CVF20 result, the total score of the NSBVA group (44.8 ± 15.6) was significantly lower than that of the control group (74.5 ± 15.5, *t* = 19.63, *P* < 0.01). According to the VF-14 result, the total score of the NSBVA group (29.8 ± 8.5) was significantly higher than that of the control group (22.9 ± 7.6, *t* = −8.71, *P* < 0.01; Table 5). Receiver operating characteristic (ROC) curve analysis showed that QOL-CVF20 reflected strong separation between the NSBVA and healthy groups, with an AUC of 0.901 (95% confidence interval 0.870-0.931), significantly greater than VF-14 (AUC = 0.738; Figure 2). Meanwhile, QOL-CVF20 could detect individuals with NSBVAs with better sensitivity and specificity than VF-14 (Table 6). QOL-CVF20 displayed specificity of 0.847 and sensitivity of 0.846, according to the maximized Youden's index (Y − index = 0.693, Table 7). Therefore, the critical value of 58.50 in QOL-CVF20 could be effectively applied for the quality of life assessment in schoolchildren with NSBVAs.

## 4. Discussion

As the subjective evaluation of a patient, QLS could make up much information about patients' social ability and psychological state, which could not be obtained by objective examination [16]. NSBVAs impaired not only binocular vision but also body function and mental and social activities of patients [8, 17]. Nowadays, the increasing incidence of NSBVAs was gradually being taken seriously [3]. In addition to concealed symptoms, the deviation of exchange and understanding between patients and doctors made the diagnose of NSBVAs more difficult. In this study, a novel QOL-CVF20 was established to quantify the quality of life in schoolchildren and could serve as early detection and clinical evaluation of NSBVAs.

Based on the theoretical concept and the entry content from WHOQOL-100, VF-14, and NEI-VFQ25, the originally designed QOL-CVF20 contained 30 entries. After a questionnaire survey of 20 schoolchildren with normal visual function and 10 schoolchildren with NSBVAs, the formal QOL-CVF20 containing 20 entries was established. During this process, the optometry test results and diagnosis results from public health experts were used as the gold standard of NSBVAs. Multiple indicators, including discrete trends, correlation coefficients, factor analysis, and discrimination validity, were applied to evaluate the entries' effectiveness. The entry would be removed if it is determined as inefficient by more than 2 evaluation indicators. By the assessment of retest reliability, Cronbach's alpha, and split-half reliability, the present QOL-CVF20 was identified to have good reliability. The significantly higher scores in NSBVA schoolchildren after therapy training and the good ES value suggested QOL-CVF20 has good response.

Predictive validity refers to the QLS ability to correctly distinguish the quality of life of the population. ROC curve is a classic method for diagnostic test evaluation and can estimate the optimal threshold for clinical practice. Our results showed that QOL-CFA20 was better than the VF-14 in terms of sensitivity, specificity, and AUC, suggesting that the QOL-CFA20 scale was better than the VF-14 scale in predicting the quality of life of schoolchildren with NSBVAs. When the score of QOL-CFA20 is 58.50, it could receive the largest Y-index. Therefore, the score 58.50 is defined as the critical value of QOL-CFA20 in the assessment of quality of life of schoolchildren with NSBVAs. These results indicated that QOL-CFA20 could accurately assess the binocular visual function of schoolchildren and provide a reference for early diagnosis of NSBVAs.

All the subjects of QOL-CVF20 were completed within the stipulated time, with 94.3% effective rate, which suggested the that this scale was acceptable and operable for schoolchildren. The main cause of invalid questionnaires was the unanswered entries, especially the item 17, “do you think your parents are concerned about you?” and item 20, “do you think your life is happy?” It might be due to their deliberate avoidance of family issues. Therefore, it should also be noticed that the privacy issue setting must be based on the confidentiality principle and mutual trust and communication between investigators and subjects.

Currently, several QLS for visual function had been applied in the world, including Activities of Daily Vision Scale (ADVS), Daily Living Tasks Dependent on Vision (DLTV), and Vison Function-14 (VF-14). Among them, VF-14, originally developed for visual function assessment in cataract patients, has been widely used to assess visual impairment in patients with various eye diseases [14, 15]. Compared with other QLS, VF-14 had many significant advantages, including small and simple items and easy to understand and answer for children [18, 19]. In the present study, through optimization of VF-14 according to the living habits of schoolchildren, QOL-CVF20 was established and received a high effective response rate in schoolchildren. Compared with original VF-14, QOL-CVF20 showed a better role in quality of life assessment in schoolchildren with NSBVAs. Therefore, QOL-CVF20 would provide evidence for early detection and diagnosis of NSBVAs in schoolchildren.

## 5. Conclusions

The present study confirmed that the novel QOL-CVF20 could reflect the life quality of schoolchildren with NSBVAs very well and was easy to operate and analyze. Through verification of various parameters, including validity, reliability, reactivity, responsiveness, and simplicity, QOL-CVF20 could be applied for NSBVAs in the clinic. However, due to limitations of human and material resources, as well as the self-assessment variability of schoolchildren life quality, there were also some deficiencies in the present QLS. Therefore, a multicenter collaborative research with a larger sample size in the future would make lots of improvements.

## Figures and Tables

**Figure 1:** The variance contribution of the common factors. (a) The eigenvalue analysis of the 4 common factors. The common factors (F1-F4) were extracted based on the principles of eigenvalues greater than 1. (b) The variance contribution analysis of the common factors. (c) The cumulative contribution analysis of the common factors.

**Figure 2:** ROC analysis of QOL-CVF20 and VF-14 on NSBVA diagnostic in schoolchildren. The AUC of QOL-CVF20 was 0.901 (95% confidence interval 0.870-0.931), and the AUC of VF-14 was 0.738 (95% confidence interval 0.691-0.785).

**Table 1:** The statistics and analysis of scores in QOL-CVF20 items.

Item	Item score	CV%	CC (score)	CC (domain)	Factor loading				SRA	SDA
					F1	F2	F3	F4		
1	3.1 ± 1.3	41.80	0.56^∗∗^	0.66^∗∗^	0.63	0.01	0.03	0.17	Y	Y
2	3.1 ± 1.3	42.33	0.60^∗∗^	0.73^∗∗^	0.76	0.01	0.03	0.00	Y	Y
3	3.1 ± 1.3	41.74	0.58^∗∗^	0.60^∗∗^	0.54	0.08	0.24	0.16	Y	Y
4	3.2 ± 1.3	41.44	0.50^∗∗^	0.56^∗∗^	0.52	0.17	0.05	0.02	Y	Y
5	3.1 ± 1.3	42.91	0.59^∗∗^	0.66^∗∗^	0.64	0.07	0.15	0.03	Y	Y
6	3.1 ± 1.3	43.41	0.56^∗∗^	0.67^∗∗^	0.70	0.02	0.01	0.02	Y	Y
7	3.2 ± 1.3	41.65	0.51^∗∗^	0.60^∗∗^	0.58	0.10	-0.05	0.09	Y	Y
8	3.1 ± 1.2	39.69	0.57^∗∗^	0.62^∗∗^	0.57	0.19	0.01	0.14	Y	Y
9	3.1 ± 1.3	41.76	0.58^∗∗^	0.71^∗∗^	0.73	0.04	-0.06	0.05	Y	Y
10	3.2 ± 1.3	42.67	0.59^∗∗^	0.69^∗∗^	0.71	0.05	0.10	-0.02	Y	Y
11	2.8 ± 1.4	49.74	0.30^∗∗^	0.85^∗∗^	-0.07	0.10	0.86	0.00	Y	N
12	2.8 ± 1.3	47.60	0.37^∗∗^	0.84^∗∗^	0.04	0.04	0.84	0.06	Y	N
13	2.8 ± 1.4	48.17	0.52^∗∗^	0.77^∗∗^	0.26	0.05	0.70	0.16	Y	Y
14	2.7 ± 1.3	46.84	0.45^∗∗^	0.84^∗∗^	0.18	0.03	0.08	0.80	Y	N
15	2.6 ± 1.2	45.90	0.34^∗∗^	0.80^∗∗^	-0.02	0.16	0.01	0.84	Y	N
16	2.6 ± 1.2	46.00	0.38^∗∗^	0.75^∗∗^	0.15	-0.03	0.11	0.69	Y	N
17	2.8 ± 1.2	45.32	0.45^∗∗^	0.79^∗∗^	0.20	0.76	0.05	-0.07	Y	N
18	2.7 ± 1.2	44.22	0.41^∗∗^	0.68^∗∗^	0.10	0.62	0.07	0.18	Y	N
19	2.7 ± 1.2	43.52	0.40^∗∗^	0.76^∗∗^	0.09	0.78	0.04	0.00	Y	Y
20	2.8 ± 1.2	43.39	0.34^∗∗^	0.74^∗∗^	0.02	0.75	0.03	0.04	Y	Y

QOL-CVF20: quality of life children questionnaire containing 20 items; CV: coefficient of variation; CC (score): the correlation coefficient for total score; CC (domain): the correlation coefficient for corresponding domain score; F1–F4: the common factors were extracted based on the principles of eigenvalues greater than 1; SRA: stepwise regression analysis; SDA: stepwise discriminant analysis; Y: yes; N: no. ^∗∗^*P* < 0.01.

**Table 2:** Comparison of QOL-CVF20 score between NSBVA and control schoolchildren.

Group	No.	Domain score				Total score
		Binocular visual function	Self-care ability	Psychological	Activity communication ability	
NSBVAs	109	26.7 ± 4.5	7.2 ± 0.7	7.8 ± 0.8	9.3 ± 1.2	49.0 ± 6.9
Control	91	34.4 ± 5.2	10.7 ± 1.1	10.5 ± 0.7	12.7 ± 1.1	69.7 ± 6.7
*t* value		-11.23	-27.26	-25.15	-20.72	-21.41
*P* value		<0.001	<0.001	<0.001	<0.001	<0.001

QOL-CVF20: quality of life children questionnaire containing 20 items; NSBVAs: nonstrabismic binocular vision anomalies.

**Table 3:** Comparison of QOL-CVF20 score from NSBVA schoolchildren before and after treatment.

Group	No.	Domain score				Total scores
		Binocular visual function	Self-care ability	Psychological	Activity communication ability	
NSBVAs	109	26.7 ± 4.5	7.2 ± 0.7	7.8 ± 0.8	9.3 ± 1.2	49.0 ± 6.9
Cured	98	31.2 ± 17.3	9.3 ± 3.7	8.9 ± 3.1	12.5 ± 2.3	61.8 ± 22.6
*t* value		-2.62	-5.81	-3.58	-12.73	-5.63
*P* value		<0.01	<0.001	<0.001	<0.001	<0.001

QOL-CVF20: quality of life children questionnaire containing 20 items; NSBVAs: nonstrabismic binocular vision anomalies.

**Table 4:** Comparison of QOL-CVF20 score from NSBVA and cured schoolchildren.

Group	No.	Domain scores				Total scores	Effect size (EZ)
		Binocular visual function	Self-care ability	Psychological	Activity communication ability		
NSBVAs	93	26.5 ± 4.9	7.1 ± 0.6	8.1 ± 1.1	9.5 ± 1.3	49.7 ± 7.2	0.53
Cured		32.3 ± 19.1	9.1 ± 2.2	8.7 ± 2.7	11.9 ± 2.1	61.4 ± 23.0	

*t* value		2.84	8.46	1.98	9.37	5.09	

*P* value		<0.001	<0.001	<0.05	<0.001	<0.01	

QOL-CVF20: quality of life children questionnaire containing 20 items; NSBVAs: nonstrabismic binocular vision anomalies.

**Table 5:** Comparison of total scores between QOL-CVF20 and VF-14.

Group	No.	Total score	
		QOL-CVF20	VF-14
NSBVAs	215	44.8 ± 15.6	29.8 ± 8.5
Control	208	74.5 ± 15.5	22.9 ± 7.6
*t* value		19.63	-8.71
*P* value		<0.001	<0.001

QOL-CVF20: quality of life children questionnaire containing 20 items; VF-14: 14-item Vision Function questionnaire; NSBVAs: nonstrabismic binocular vision anomalies.

**Table 6:** Forecast indicators of QOL-CVF20 and VF-14.

Scale	Sensitivity (%)	Specificity (%)	Positive predictive values (%)	Negative predictive values (%)	AUC
QOL-CVF20	84.6	84.7	85.0	84.2	0.901
VF-14	87.9	51.0	64.1	79.7	0.738

QOL-CVF20: quality of life children questionnaire containing 20 items; VF-14: 14-item Vision Function questionnaire; AUC: area under curve.

**Table 7:** The sensitivity and specificity corresponding to the critical value of QOL-CVF20.

Critical value	Sensitivity	Specificity	1 − specificity	Youden's index
56.00	0.880	0.800	0.200	0.680
57.50	0.865	0.823	0.177	0.688
58.50	0.846	0.847	0.153	0.693
59.50	0.837	0.851	0.149	0.688

QOL-CVF20: quality of life children questionnaire containing 20 items.

## Data Availability

The data used to support the findings of this study are available from the corresponding author upon request.

## Supplementary Materials

Supplementary Materials Table S1: the detailed content of QOL-CVF20.
